This article has been retracted.

# CNN-LSTM Hybrid Real-Time IoT-Based Cognitive Approaches for ISLR with WebRTC: Auditory Impaired Assistive Technology

**DOI:** 10.1155/2022/3978627

**Published:** 2022-02-21

**Authors:** Meenu Gupta, Narina Thakur, Dhruvi Bansal, Gopal Chaudhary, Battulga Davaasambuu, Qiaozhi Hua

**Affiliations:** ^1^Department of Computer Science and Engineering, Chandigarh University, Punjab, India; ^2^CSE Department, Bhagwan Parshuram Institute of Technology, New Delhi, India; ^3^Department of Electrical and Electronics Engineering Department, Bharati Vidyapeeth's College of Engineering New Delhi, New Delhi, India; ^4^Bharati Vidyapeeth's College of Engineering, New Delhi, India; ^5^Department of Electronics and Communication Engineering, School of Engineering and Applied Sciences, National University of Mongolia, Ulan Bator, Mongolia; ^6^Computer School, Hubei University of Arts and Science, Xiangyang 441000, China

## Abstract

In the era of modern technology, people may readily communicate through facial expressions, body language, and other means. As the use of the Internet evolves, it may be a boon to the medical fields. Recently, the Internet of Medical Things (IoMT) has provided a broader platform to handle difficulties linked to healthcare, including people's listening and hearing impairment. Although there are many translators that exist to help people of various linguistic backgrounds communicate more effectively. Using kinesics linguistics, one may assess or comprehend the communications of auditory and hearing-impaired persons who are standing next to each other. When looking at the present COVID-19 scenario, individuals are still linked in some way via online platforms; however, persons with disabilities have communication challenges with online platforms. The work provided in this research serves as a communication bridge inside the challenged community and the rest of the globe. The proposed work for Indian Sign Linguistic Recognition (ISLR) uses three-dimensional convolutional neural networks (3D-CNNs) and long short-term memory (LSTM) technique for analysis. A conventional hand gesture recognition system involves identifying the hand and its location or orientation, extracting certain essential features and applying an appropriate machine learning algorithm to recognise the completed action. In the calling interface of the web application, WebRTC has been implemented. A teleprompting technology is also used in the web app, which transforms sign language into audible sound. The proposed web app's average recognition rate is 97.21%.

## 1. Introduction

A system of communication through which humans share or express their views, thoughts, ideas, and expressions can be defined as language. Language plays a vital role in connecting individuals to their society and surroundings. India is popularly known as a land of many tongues, where as many as 22 languages and several dialects are spoken natively. Apart from these languages, the Indian sign language (ISL) came into existence since 2001 at Ali Yavar Jung National Institute for the Hearing Handicapped (AYJNIHH) in Mumbai for the people who are hearing and listening impaired. The indications used in sign language differ by area in a country that is linguistically and culturally varied, such as India. ISL is a set of visual signals, hand cues, and gadgets used by deaf and mute people for communicating with one another and to connect them with this society. ISL is the major means of exchanging emotions and notions for the deaf and mute community to connect with commons in India.

### 1.1. Problem Statement

As stated by World Health Organization's 2011 statics, approximately sixty-three million individuals in India are either completely or partially deaf, with at least 5 million of them being children [1]. As per the WHO, 466 million people worldwide suffer from speech and hearing impairments, with 34 million of them being teens. According to estimates, this number might rise to over 900 million by 2050 [2].

Such people who are mute and deaf feel lonely in this world of infinite population, and these feelings affect them physically and mentally. To sustain these challenges, IoMT has provided an important platform for advancement in technical fields related to healthcare as identification of sign languages acts as a beginning in assisting persons with hearing impairment in overcoming social stigma, unemployment, and lack of formal education. It is past time for us to provide a hand in breaking down this barrier of silence. The least advancements have been made in Indian Sign language Recognition (ISLR). Hence, through this research, an interface will be developed that will be beneficial for the Indian community of the impaired. Real-time translation of ISL is not practiced yet.

Through this manuscript, the authors want to acknowledge the needs of persons with hearing and listening difficulties that had been overlooked and predict the progress of sign language research. This article targets this problem by introducing a novel and robust system (web app) based on ISL to subtitle converter video calling applications that will help a hearing and listening impaired person talk with others.

### 1.2. Contribution

Higher response time has always been a subject of debate. Thus, attempts will be made to reduce the response time so that it will be nearly negligible. In this article, instead of conventional techniques on which the ISLR normally relies, an attention-based 3D-CNNs and LSTM for ISLR has been proposed. In the realm of human–machine interaction, gesture detection and hand postures tracking are useful approaches.

Identifying the hand and its location or orientation, extracting some relevant characteristics, and using an appropriate machine learning algorithm to recognise the executed action are all steps in a standard hand gesture recognition system. For building the web app [3], WebRTC has been implemented in the calling interface and python has been used for training data. This solution deals with the detection and recognition of hand gestures and then converting them into text in the form of subtitles or captions on the screen during real-time communication. The app is based on artificial intelligence that requires user input as sign language. The web app also uses a teleprompting system that converts sign language into audible sound [4–6]. There are numerous advantages of such systems on the societal level.

- They can be used for assisting hearing and speech impaired pupils in their early phases of growth and provide them with a crystal-clear picture of communication
- The process of learning and teaching can be enhanced
- They provide the language adaptability that eliminates the need for the impaired to acquire a new language and vice versa, resulting in a unified system that can be utilized by everyone [7–10]

This article focuses on peer-to-peer networks. Once peer 1 starts calling to peer 2, then from the very first, the signal from peer 1 hits the WebRTC interface by peer 2 server (TURN server and STUN server). Here, WebRTC gateway has been used for video calling, as it makes the process very fast via a peer-to-peer connection. This article is further divided into various segments: Section 2 discusses the view of several researches on ISL and hand gestures. Section 3 discusses the data collection, proposed methodology, and model formulation. Section 3 has shown the various matrices and methods applied in this work for analysis. Section 4 discusses the assessment of training/testing outcomes using confusion matrices for the systems used. Finally, this article is concluded in Section 5 with its future scope.

## 2. Literature Review

According to census 2011, it is a fact that around 63 million people suffer from hearing and listening problems and they are considered to be nothing by the people of this society [2]. Creating awareness among the people regarding sign language is of high importance, and one of the ways of creating such awareness is to promote sign language education among the children at primary, secondary, and higher education levels. Many researchers have already done a lot of work in this field for different sign languages such as American sign language (ASL), Italian gestures [11–14], Chinese sign language (CSL), and Arabic sign language (ArSL) as sign language varies from region to region. Thus, there is a lack of a standardized dataset of sign languages. Previous works related to sign language were mainly done based on esteemed studies [15–18], where hand detection algorithms were separated into two classifications: appearance-based and model-based.

To enable hand gesture identification, an appearance-based technique has been used to detect fingertips. A neural network-based system distinguishes continuous hand positions from grey-scale video pictures in this method. On the other hand, in the model-based approach, El-Sawah et al. [19–22] calculated the likelihood of skin colour observation using a histogram [23–25]. Artificial Neural Networks (ANNs)/learning-based methodologies [26–29], fuzzy logic, and genetic algorithm-based techniques [19] have all been presented as solutions for hand detection. Dardas and Georganas [30] used the BOF technique and a multiclass SVM classifier to create a hand gesture detection and identification system. They created a syntax that yields gesture commands that may be used to control apps. Under varying conditions, their system may produce adequate real-time performance along with high-classification accuracy. However, their system is only capable of detecting and tracking static postures. Their grammar could not make sentences out of their immobile postures. Moreover, appearance-based methods, depth of field and hand posture information, may limit the system's versatility.

Tripathi [31] suggested a continuous (ISL) hand gesture system that uses both hands to execute any gesture and uses a gradient-based key frame extraction method to separate continuous sign language gestures into sequences of signs and remove uninformative frames. Orientation histogram (OH) is used to extract additional features from preprocessed motions, while principal component analysis (PCA) is used to tune the parameters of the features extracted after OH. In [32], the authors presented work on German and Danish sign language using weakly supervised learning for continuous Sign Language. Neverova et al. [33] offered a multiscale classification technique based on colour, depth data, and custom posture descriptors. To extract visual signals for arm areas, CNNs and 3D-CNNs have been used. In [34], the authors proposed a novel framework for multimodal gesture recognition using deep dynamic neural networks (DDNN) based on HMM by different input parameters. In [35], authors used 3D-CNNs to retrieve spatiotemporal features from streaming videos using colour, depth, and optical flow data. R. Cui. et al. [36] proposed a system that uses a DNN to transcribe videos of SL phrases into sequences of ordered labels. In [37], A. Mittal et al. proposed a modified LSTM model for consecutive sequences of gestures or continuous SLR, which identifies a series of connected gestures and is evaluated with 942 ISL sign phrases using 35 distinct words. On individual sign words, there was an average accuracy of 89.5 percent. X. Ma and E. Hovy [38] created a sequence labelling algorithm using a mixture of bidirectional LSTM, CNN, and CRF. In [39], the author has discussed action recognition using videos by applying deep bidirectional LSTM (DB-LSTM). In [40], the authors proposed an SLR framework, which is majorly based on CSL using CHMM and bidirectional LSTM. In [41], following the hybrid method to sign language recognition, powerful CNN-LSTM models in each HMM stream are embedded. They put the classifiers through their paces on three publicly accessible datasets: challenging real-life German sign language with over 1000 classes, full phrase-oriented lip reading, and articulated hand shape recognition on a fine-grained hand form taxonomy with over 60 unique hand forms. Joy et al. [4] talked about Sign Quiz, a low-cost web-based fingerspelled sign learning tool for ISL that uses a deep neural network for automated sign language identification. In [42], Daniel et al. demonstrated a method for searching huge video collections for clips that reflect a natural language query expressed as a phrase.

The abovementioned analyses are the opinions of different researchers about the use of different techniques and deep learning frameworks in the field of gesture recognition under varying conditions of several kinds of sign language, whereas this research is mainly focused on ISL. In contrast to previous studies, a three-dimensional CNN-LSTM hybrid-based solution that operates in real time on a web browser has been created here. This can directly be incorporated with the idea of IoMT to help uplift individuals in the challenged community. Sections 3 and 4 discuss the detailed descriptions of the proposed method and its analysis.

## 3. Materials and Methods

The proposed analysis started from training a corpus so that this system could intelligently predict a sign. For this purpose, the author tried working on different available datasets so that features, namely, matching points, edges, nodes, and movement of gestures could be identified. However, the hurdle that majorly blocked the path of machine training was firstly the lack of abundant characters and words from the dictionary of India. Secondly, even though some of the datasets were available with all the necessary and sufficient words, they were collected for purposes that were completely different than the author's requirements, i.e., communication between the impaired and commons. Lastly, if the available datasets were defeating the above hurdles, then the biggest of all problems come into existence; that is, the quality of the image was not appropriate to feed into a CNN-LSTM [43] network; however, the author compiled this specific algorithm for the following reasons:

- If the feature matrix of the gesture was fed as the corpus, it would have caused as much delay as of 5 times, as the feature matrix need to be converted into an image and vice versa
- The best algorithm for processing images for machine learning is found to be the CNN-LSTM as classic CNN is necessary and sufficient for a single image and LSTM can hold the memory of the last processed corpus and eligible for multiple images

### 3.1. Dataset Used

The goal of this work is to analyse and recognise various alphabets, numbers, and words using a collection of pictures of sign. The database contains a variety of pictures, each of which was taken under different lighting and with distinct hand orientations. This system has been trained to achieve excel levels and hence attain decent results with such a diverse data collection. This work used the primary dataset, as shown in Figure 1. The defined notation for ISL number (0–9) and alphabets (A–Z), which consists of a total of 42000 images, from which 1200 images were of each sign. Then, preprocessing of the images of the dataset, i.e., Image Acquisition, was done.

The images captured by the webcam required preprocessing before going to the next step, as presented in Figure 2.

In the preprocessing step, background subtraction [44] and cropping of hand are done. Then, the image is transformed into a grey-scale image as the RGB colour image contains an extra matrix of colours, i.e., [R, G, B] that is not necessary for any edge detection techniques in gesture detection). After that, feature extraction, orientation detection (There are several features, or relevant spots on an item, that can be extracted to generate a “feature” description of the object for every object. The main points are then given a consistent orientation depending on local image characteristics.), and gesture recognition is done through a convex hull algorithm.

### 3.2. Preprocessing of Dataset

After applying the stages of the algorithm, processing of the image was done as shown in Figure 3. The preprocessing steps include segmentation, morphological processing, and training of deep convolved neural network to analyse the best performance of the proposed algorithm. Steps of the algorithm are as follows [45].

#### 3.2.1.  Gray Scale Conversion of Image

A technical misnomer for grayscale imaging is often used as “black and white imaging.” The only hues available in genuine black and white, commonly known as halftone are pure black and pure white. The appearance of grey shading in a halftone image is achieved by displaying the image as a grid of white dots on a black backdrop (or vice versa), with the sizes of the individual dots corresponding to the virtual luminance of the grey in their immediate vicinity. The halftone method is frequently used in the printing of photos in newspapers. The illumination levels of the hues, namely, Red (R), Green (G), and Blue (B) components, are each expressed as a value from decimal 0 to 255 or binary 0x00 to 0xff in the case of transmitted light (for instance, the picture on a computer screen). For each RGB [46] grayscale pixel picture, R = G = B. The brightness levels of the primary colours are a major factor that influence the lightness of the grey in direct proportion. Black is depicted as B = R = G = 0 or B = R = G = 0x00, and white is denoted by B = R = G = 255 or B = R = G = 0xff. This photographic method is known as 8-bit grayscale because the binary representation of the grey level has 8 bits. It is a collection of grayscale images with no discernible colour. The darkest attainable shade is black, which is the entire disappearance of transmitted or reflected light, while the lightest possible shade is white, which is the total transmission or reflection of light at all optical wavelengths. As a result of the aforementioned factors, first, the sign language pictures are converted into grayscale images in this preprocessing phase.

#### 3.2.2. Noise Removal Using High-Pass Filter

Proceeding with that, the grayscale image acquisition is given as a parameter to the high-pass filter. The most common sharpening procedures start with a high-pass filter. When contrast is increased between adjacent regions with a minor change in brightness or vice versa, image sharpening occurs. It is prone to preserving high-frequency data while reducing low-frequency data in a picture. The origin of this filter is formulated to enhance the brightness of the center pixel as compared to its vicinity pixels. The origin array generally structures a single + ve value at its center, which is totally encapsulated by -ve values.

#### 3.2.3. Application of Median Filter for Image Quality Enhancement

It is typically desirable in image processing to be able to do some form of noise removal on an image or input. This filter is a type of nonlinear digital filter that is frequently implemented to eliminate noise. As a result, noise reduction is a common preprocessing way to enhance the outcomes of subsequent processing (e.g., edge detection on an image). Because it retains edges while eliminating noise, median filtering is frequently employed in digital image processing under specific conditions. The median filter's primary idea is to go bit by bit through the signal, exchanging each bit with the median of neighboring bits. The “frame” is a swatch of neighbors that moves across the whole signal, entry by entry. For 1D inputs, the most obvious frame is the barely introducing and following entries, but for 2D (or more dimensional) signals like pictures, more complicated window shapes are likely (such as “box” or “cross” patterns). It is worth noting that the median for an odd number of entries in a window is straightforward to define as it is just the central value after all the items in the window have been sequentially sorted. If the number of items in a window is even, there are many medians to choose from. The image quality can be enhanced by using this filter.

#### 3.2.4. Morphological Operations for Image Feature Extraction

It is an iteration of nonlinear process associated with the form or morphology of qualities in a picture. Morphological processes are the greatest match for the processing of binary pictures since they rely only on the relative arrangement of pixel values rather than their numeric value. It may be used on grayscale pictures if their light transfer functions are unknown, resulting in insignificant absolute pixel values. Morphological methods reveal an image that has a little shape known as a structuring element. The structuring element is applied to the image at the tiniest possible boundaries and compared to the pixels in the surrounding area. Some processes examine whether the element “fits” in the environment, while others examine at how likely it is to strike or intersect with the environment: if the inspection is successful at that point within the picture to be processed, this operation on a Boolean image creates a replacement Boolean image in which the pixel has a nonzero result. The structuring element could be a small binary image, i.e., a little matrix of pixels, each with a price of zero or one:

- The dimensions of the matrix define the dimensions of the structuring element
- The shape of the structuring element is defined by the pattern of ones and zeros within the matrix
- The mother of the structuring element is sometimes one in every of its pixels, although usually, the seed is the extra structuring element

#### 3.2.5. Threshold Segmentation Computation

The segmentation block now receives the feature extracted picture, which is divided into sets of segments that together cover the whole image. This is one of the major steps led in this algorithm as most of the currently available methods directly introduced present the dataset as the training input to the classifier. Segmentation has been applied to the feature extracted image, hence easing the region of interest to make it more meaningful and easier to study. Otsu's method (maximum variance) has been used for threshold segmentation computation.

### 3.3. Proposed Model

Compared to networks with fully connected layers, the CNN, which is also known as “ConvNet,” has a deep perceptron structure and a remarkable capacity to generalise. It is capable of learning very intellectual characteristics and identifying the items effectively. The following are the rationale why CNN is preferred above other traditional models. Firstly, the notion of leveraging the concept of weight sharing is to minimise the number of parameters that need to be trained, resulting in greater generalisation, which has piqued researcher's curiosity. This classifier can be learned smoothly with fewer parameters and avoids overfitting. Secondly, the classification step is combined with the feature extraction stage, both of which are based on learning. At last, we can conclude that the massive networks utilizing generic models of ANN are significantly more complex than those implemented in CNN. Due to their exceptional performance, CNNs are widely utilized in a variety of areas, including image stratification, object identification, facial expression identification, vehicle recognition, and recognition of voices.

#### 3.3.1. Proposed Model Architecture

The standard ANN model comprises linearization SISO (single-input single-output) and many hidden layers. A specific neuron takes an input vector A and performs a function F on it to create an output vector B [47]. The weighed vector that was created may now be utilized to execute picture classification. There is a substantial quantity of literature on pixel-based picture categorisation. Contextual information, such as the image's shape, gives better results or outperforms. CNN is a model that is gaining popularity due to its capacity to classify objects and handle the relevance of accounting data. A convolution layer, a pooling layer, an activation function, and a fully linked layer are the four aspects of the CNN model. The connection of layers in the proposed model is shown in detail in Figure 4.

#### 3.3.2. Performance Analysis of the Proposed Model

In this section, the proposed model used in this work is described based on performance are as follows.

*(1) Convolutional Layer*. The system receives an image to be categorised, and the envisaged class label is calculated using feature extraction from the picture. The local connection between an individual neuron in the next layer and certain neurons in the preceding layer is known as the receptive field. The input image's local characteristics are retrieved via receptive field analysis. This field of a neuron linked with a certain area in the preceding stage is represented by a weight vector that remains constant at all places on the plane, where the plane refers to the neurons in the next layer. Because the weights of the neurons in a plane are identical, comparable characteristics appear at various points in the input data. The feature map is created by sliding the weight vector, also known as the filter or kernel, across the input vector. Convolution operation refers to the process of moving the filter horizontally and vertically. This procedure collects the N range of attributes from the input picture in a single layer, resulting in N filters and N feature maps. The range of training parameters is considerably decreased due to the phenomena of the local receptive field.

*(2) Pooling Layer*. Once a feature has been recognised, its specific position becomes less important. As a result, the pooling or interlayer comes after the convolution layer. The main benefit of adopting the pooling approach is that it significantly lowers the range of training parameters while also introducing translation invariance. A frame is chosen for the pooling [28] procedure, and the input components inside that frame are sent via a pooling function.

*(3) Fully Connected Layer*. In traditional models, the fully connected layer is identical to the fully linked network. The output of the first phase (which involves repeated convolution and pooling) is sent into this layer, which computes the dot product of the weight and the input vector to get the result. Gradient descent [47] lowers the cost function by calculating the cost over an entire training dataset and updating the parameters just once every epoch. It produces global minima, but if the training dataset is enormous, the time it takes to train the network has tremendous growth. Speculative gradient descent was used to supplant this method of cost function reduction.

*(4) Activation Function*. There is a heavy emphasis on the sigmoid activation function in traditional machine learning methods. Because of two key considerations, the usage of the Rectified Linear Unit (ReLU) has proven to be superior to the former in terms of introducing nonlinearity. At the beginning, the computation of the partial derivative of ReLU is simple. Furthermore, saturating nonlinearities such as sigmoid are taken into account during training time. On the other hand, the ReLU function does not allow gradients to be exterminated. However, when a significant gradient flows through the network, the effectiveness of ReLU worsens, and updates in weight lead the neuron not to be triggered, resulting in the Dying ReLU situation, which is a common occurrence.

The basic LSTM cannot easily represent input with spatial structure, such as pictures. The CNN-LSTM architecture is built particularly for classification predictive issues [48] using spatial inputs such as pictures or clips. The CNN layers for feature extraction on input data are coupled with LSTMs to provide sequence prediction in the CNN-LSTM structure, as shown in Figure 5.

CNN LSTMs were created to solve visual time series prediction issues and generate textual descriptions from picture sequences, in particular, the following issues:

- Activity recognition: using a sequence of pictures to generate a written description of an activity
- Image explanation: the process of creating a written description for a single image
- Video explanation: creating a textual description of a picture sequence

The LSTMs [49] referred to here that employ a CNN as a front end as “CNN-LSTM” were initially referred to as a [50] long-term recurrent convolutional network or LRCN model. The task of creating textual descriptions of pictures is accomplished using this framework. The employment of a CNN that has been pretrained on a difficult picture classification job and then repurposed as a feature extractor for the caption producing issue is crucial. CNNs have also been utilized as feature extractors for LSTMs on audio and textual input data in voice recognition and natural language processing challenges. This structure is suited for the following types of problems:

- Input that has spatial structure, such as the 2D structure of pixels in a picture or the 1D structure of phrases, section, or text
- Inputs having temporal structure, such as the sequence of pictures in a clip or phrases in text, or outputs with temporal structure, such as words in a text content, are required

In this context, a 2D convolutional network comprising of Conv2D and MaxPooling2D layers is arranged into a stack of the necessary depth. The polling layers will integrate or abstract the perception of the Conv2D, which analyses snapshots of the picture, such as signs. Max-Pooling 2D divides the processing into 2 × 2 blocks, resulting in an 8 × 8 integration. The flatten layer will take the single 8 × 8 element map and convert it to a 64-element vector, which may then be processed by another layer, such as a dense for prediction output. Only a single image may be processed by the CNN model, which converts input pixels into an internal matrix or vector form.

This procedure must be repeated over numerous pictures in order for the LSTM to build up an internal state and update weights using backpropagation through time (BPTT) throughout a succession of internal feature vectors of input images. When utilizing an existing pretrained model like Visual Geometry Group (VGG) for feature extraction from pictures, the CNN could be helpful. The author may want to train the CNN by backpropagating error from the LSTM throughout several input pictures to the CNN model if it is not already trained. In all of these situations, a simple CNN model and a succession of LSTM models, one for each time step, are theoretically present. Here, the CNN model is applied to each input picture and sends the output to the LSTM in a single time step. This may be accomplished by encasing the whole CNN input model (one or more layers) in a dense layer. This layer provides the intended result of repeatedly applying the same layer or layers. In this example, it was applied many times to various input time steps, resulting in a set of “image judgement” or “image features” for the LSTM model to operate with. The working of the proposed methodology has been shown in Figure 6.

#### 3.3.3. Training of the Model Based on Collected Data

Once the set of images was converted into the textual description (that is, key-value pairs based on .xml schema) after training, the problem domain converts to store that bag of trained words to be translated while communicating over the web channel. Thus, once trained using Conv2D nets followed by Maxpooling2d, Activation, and dense layers, the bag of words are stored as h5py or json schema, as the JSON format is easily accessible in real time because it does not need any extra parsing engine rather than the WebRTC itself. Thus, the approach of training and prediction in contrast to the conventional methods, i.e., in a single source, was changed to training for a single time of the seed and stores the seed information in the dictionary based on JSON schema, which is finally embedded with the real-time communication STUN server. Once the dictionary was embedded with the STUN server, it could be easily mapped with a processing file based on natural language processing to translate the sign features into perfect words. The natural language process step considers the dictionary (created earlier) as the elementary dataset and bag of words to covert a sequence of signs into words and sentences (real-time captioning of the image)[51].

### 3.4. Proposed Algorithm

**Step 1 .**

Image preprocessing, i.e., image = Y

**Step 2 .**

Combine the picture with a pretrained model's input

**Step 3 .**

Retrieve the output of the provided model's last convolution layer

**Step 4 .**

Reduce the number of *n* dimensions to n-1 to flatten them

**Step 5 .**

Apply different layers of CNN

Various CNN layers have been performed in detail here, as indicated in equations (1)–(11).

(i) Padding (Conv2d): the padding width should be calculated using the formula below, where *p* is the padding and *f* is the filter dimension (f ∈ odd).
  (1) $$\begin{array}{c} p=\frac{f-1}{2}. \end{array}$$
(ii) Forward propagation: it is divided into two stages. To begin with, it computes the intermediate value Z, which is generated by convolution of the preceding layer's input data with the W tensor (including filters) and further adds bias b. In addition, it involves applying a nonlinear activation function on intermediate value (activation ⟶ g).
  (2) $$\begin{array}{c} Z^{\left[l\right]}=W^{\left[l\right]}\cdot A^{\left[l-1\right]}+b^{\left[l\right]};A^{\left[l\right]}=g^{\left[l\right]}\left(Z^{\left[l\right]}\right). \end{array}$$
(iii) Max-pooling: the proportions of the output matrix may be determined using the following formula, taking padding, and stride into consideration:
  (3) $$\begin{array}{c} n_{\text{out}}=\left[\frac{n_{\text{in}}+2p-f}{s}+1\right]\;. \end{array}$$
The first and most essential criterion is that the filter and the picture to which it is applied must have a similar numeral of channels. If one wants to apply many filters on the same picture, then each one is independently convoluted; the outcomes were stacked one on top of the other and then merged into a whole. The proportions of the received tensor (as 3D matrix had been named) satisfy the following equation: *n* ⟶ picture size, *f* ⟶ filter size, nc ⟶ number of channels in the image, *p* ⟶ used padding, *s* ⟶ used stride, nf ⟶ number of filters.
  (4) $$\begin{array}{c} \left[n,n,n_{c}\right]*\left[f,f,n_{c}\right]=\left[\left[\frac{n+2p-f}{s}+1\right],\left[\frac{n+2p-f}{s}+1\right],n_{f}\right]. \end{array}$$
(iv) Partial derivative of the cost function is as follows:
  (5) $$\begin{array}{c} dA^{\left[l\right]}=\frac{\partial L}{\partial A^{\left[l\right]}}\;;dZ^{\left[l\right]}=\frac{\partial L}{\partial Z^{\left[l\right]}}\;;dW^{\left[l\right]}=\frac{\partial L}{\partial W^{\left[l\right]}};\;db^{\left[l\right]}=\frac{\partial L}{\partial b^{\left[l\right]}}. \end{array}$$

After applying chain rule,

(6) $$\begin{array}{c} dZ^{\left[l\right]}=dA^{\left[l\right]}*g^{\prime }\left(Z^{\left[l\right]}\right). \end{array}$$

**Step 6 .**

Apply activation

(i) Sigmoid activation function: A sigmoid function has a range of 0 to 1. This implies that regardless of the input value, the output will always be inside the range (0, 1). A Sigmoid function is commonly employed in binary classification issues, so both convolutional and fully connected layers have been applied.
  (7) $$\begin{array}{c} f\left(x\right)=\frac{1}{1+e^{-x}}. \end{array}$$
(ii) Linear transformation equation is as follows:
  (8) $$\begin{array}{c} Z\;=\;W^{T}.X\;+\;b. \end{array}$$
(iii) Leaky ReLU: here, the ReLU activation function has been specified as a very tiny linear component of *x* rather than as 0 for negative values of inputs(*x*). This activation function's formula is as follows:
  (9) $$\begin{array}{c} f\left(x\right)=\left(0.01{}^{*}x\;,\;x\right) \end{array}$$

If it receives a positive input, it returns *x*; if it receives a negative input, it returns a very small value equal to 0.01 times *x*. As a result, it also produces an output for negative values. By making this minor change, the gradient on the left side of the graph becomes nonzero.

**Step 7 .**

Apply Softmax function

In general, not even one final figure is produced by the neural network. However, it is essential to decrease these values to integers from zero to one, which indicates each class's probability. The Softmax function plays this role:

(10) $$\begin{array}{c} \sigma \;:R^{K}⟶{\left(0,1\right)}^{K}, \end{array}$$

(11) $$\begin{array}{c} \sigma {\left(z\right)}_{j}=\frac{e^{zj}}{\sum_{k=1}^{K}e^{z_{k}}}\;for\;j=1,\ldots .,K. \end{array}$$

**Step 8 .**

Applying LSTM

After applying CNN, LSTM has been implemented. Results have been formulated as discussed in equations (12)–(17).

(i) The LSTM gate equations are as follows:
  (12) $$\begin{array}{c} i_{t}=\;\sigma \left(w_{i}\left[h_{t-1},\;x_{t}\right]+b_{i}\right), \end{array}$$
  (13) $$\begin{array}{c} f_{t}=\;\sigma \left(w_{f}\left[h_{t-1},x_{t}\right]+\;b_{f}\right), \end{array}$$
  (14) $$\begin{array}{c} o_{t}=\;\sigma \left(w_{o}\left[h_{t-1},\;x_{t}\right]+\;b_{o}\right), \end{array}$$
where *x*_*t*_ ⟶ input at current timestamp,*h*_*t*−1_⟶ output of the previous Istmblock(at timestamp *t*  −  1), *w*_*x*_ ⟶ weight for the respective gate(*x*)neurons,*σ* ⟶ represents sigmoid function,*f*_*t*_ ⟶ represents forget gate,*i*_*t*_ ⟶ represents input gate,and *b*_*x*_⟶ biases for the  respective gates(*x*).
(ii) The equations for the cell state, candidate cell state, and final output are as follows:
  (15) $$\begin{array}{c} \tilde{c_{t}}=\tanh\tanh\;\left(w_{c}\left[h_{t-1},\;x_{t}\right]+\;b_{c}\right), \end{array}$$
  (16) $$\begin{array}{c} c_{t}=\;f_{t}*\;C_{t-1}+\;i_{t}*\tilde{c_{t}}, \end{array}$$
  (17) $$\begin{array}{c} h_{t}=\;o_{t}*\;\tanh\tanh\;\left(c^{t}\right), \end{array}$$
where *c*_*t*_⟶ is the cell state (memory) at timestamp (t). $\tilde{c_{t}}\;⟶\;$ represents candidate for cell state at timestamp (*t*).

## 4. Results Formulation

In result analysis, the findings were then compared to decide which model was the best. Although the model's accuracies are quite good, evaluation has been recommended by the performance with future dataset updates. Due to a lack of data, the model has been trained on only 33600 samples and tested on 8400 [52].

### 4.1. Metrics Used

The suggested model was tested using several metrics such as precision, recall, *F*1 score [53] and its accuracy, sensitivity, and specificity [54]. The suggested model was assessed using various metrics such as precision, recall, *F*1 score, and accuracy, sensitivity, and specificity, as stated in the following equations:

(18) $$\begin{array}{c} \text{precision}=\frac{\text{true positive}}{\text{true positive }+\text{ false negative}}\text{,} \end{array}$$

(19) $$\begin{array}{c} \text{recall }=\frac{\text{true positive}}{\text{true positive }+\text{ false negative}}\text{,} \end{array}$$

(20) $$\begin{array}{c} \text{F}1\text{ score }=2*\frac{\text{precision }*\text{ recall}}{\text{precision }+\text{ recall}}\text{,} \end{array}$$

(21) $$\begin{array}{c} \text{accuracy }=\;\frac{\text{true positive }+\text{ true negative}}{\text{true positive }+\text{ false negative }+\text{ true negative }+\text{ false positive}}\text{.} \end{array}$$

The dataset's feature was extracted and trained using multiple layers of the CNN method, which was then coupled with LSTM to assist sequence prediction, as it aids in the generation of textual descriptions from a sequence of pictures. Here, CNN acts as encoder, whereas LSTM is acting as a decoder. Results of CNN and LSTM are evaluated and discussed in detail based on precision, *F*1-score, and recall of training and testing data, respectively, as shown in Table 1.

Precision indicates the promotion of positive identifications that were actually correct. A model that produces no false positives has a precision of 1.0. Recall indicates the proportion of actual positives that were correctly classified. A model that produces no false negatives has a recall of 1.0, whereas one score is the combination of precision and recall. A perfect model achieves an *F*1 score of 1.0. For a total of 35 labels [55], here, in which 0 to 9 depicts numbers (0 to 9) and 10 to 34 labels depict the alphabets from (A to Z), all scores based on evaluation metrics are shown and analysed in Figures 7(a) and 7(b) of training and testing, respectively. Here, 240 samples of each label were taken into account for this classification report.

Figure 8 shows the overall comparison of scores based on evaluation metric parameters for training and testing by applied model.

This model contains 35 target classes to measure the classification model's performance, resulting in confusion metrics of 35 × 35. Essentially, it compares the actual targeted labels to the predicted labels predicted by the suggested model.  Figure 9 shows the confusion matrix obtained from the true labels and predicted labels.

Categorical cross-entropy is a loss function used in multiclass classification problems. These are problems in which an example may only belong to one of several potential categories, and the model must determine which one it is. Its formal purpose is to measure the difference between two probability distributions. Here loss is calculated by using the categorical loss function stated as in the following:

(22) $$\begin{array}{c} L_{CE}=\;-\sum_{i=1}^{n}t_{i}\log\log\;\left(p_{i}\right),\;\text{ for }n\text{ classes,} \end{array}$$

where *t*_i_ is the truth label; *p*_i_ is the Softmax probability for *i*^th^ class.

Classification accuracy is one of the measures used to assess your model's performance. It can be stated as follows:

(23) $$\begin{array}{c} \text{accuracy}=\frac{\text{no. of correct predictions}}{\text{total predictions}}. \end{array}$$

In Figure 10(a), cross-entropy loss depicts the training loss for the custom model as it decreases over time, whereas from Figure 10(b), the classification accuracy depicts the accuracy of the custom model as it is enhanced over time.

### 4.2. Communication between Sign and a/v Channel

Considering real-time communication, it will take time to show subtitles after converting from signs. WebRTC signal is only triggered once at the server and it starts communication serverless. This is known as signal communication and data of call are not getting stored in any database, so it maintains the privacy of users. First, images have been captured from camera one of client one and then preprocessing of data is done, which includes cropping of his hands and background subtraction and other processing of data of images. Then, all these data of client one, which is in ISL, are passed through video calling by creating a request on WebRTC, then data are compared from h5.py where it will get recognised by the model of image classification and gets converted in the form of subtitles and gets converted into audio format to the client and subtitles will appear on client 2's screen. Once all the training is done, namely, sign (image), subtitle (bag of words), and audio (speech), the entire system is ready to use. Any data from a peer causes a trigger in the TURN server. Once the trigger is achieved, it creates another peer known as real-time peer, which starts handling the rest of the communication process. The gateway embeds contain the translator created in the above step after training the model. The translator detects hand in a sequence and if a hand is detected, an async-await process starts to resolve the problem for checking in the dictionary for the valid character, number, or word. Once the problem is resolved, the subtitle is provided to the text-to-speech [33] synthesizer and the process succeeds. If the problem is not resolved, it awaits till a sign is detected. The detailed architecture is shown in Figure 11.

Results and evaluation of video calling web app “Dhruvi calling Dhruvi” are shown in Figure 12 where Figure 12(a) indicates letter “X,” 12(b) indicates letter “B,” and 12(c) indicates number “3,” respectively.

## 5. Conclusion and Future Scope

This model implements a module that can be used as a common media of idea transaction between impaired and commons. The idea of hybrid CNN-LSTM was applied because the convolutional neural network is efficient for the training of one single-input image, whereas LSTM with a convolutional neural network is used to pass a CNN model into LSTM so that it can be passed through WebRTC, which can be used as a kernel. The accuracy of training was found to be 81.58%. The accuracy of testing the kernel was found to be 99.58%. Once the kernel was trained, the neural network was converted into schema so that it can be accessible by WebRTC for communication. Python TTS library is used to generate voice from subtitles that originate from images. It could basically detect all English words and digits from 1 to 9. However, due to the lack of dataset belonging to 0 and punctuation, the current interface has a few issues that can be resolved in the next modules. If better datasets are accessed in the near future, the training accuracy can be amplified. This web app will also help in the education sector for such persons. The proposed architecture acts as an interface for video calling, which can be further implemented as a teleprompter. The device can be fabricated in wearables so that a normal person can understand the sign language just after wearing it. The device can be trained in other sign languages so that it will not be a locale to Indian Market. It is expected that the system and the results presented in this article would provide an example for future work based on the Indian sign language.

## Figures and Tables

**Figure 1:** Samples of Indian sign language dataset.

**Figure 2:** Creation of Indian sign language dataset.

**Figure 3:** Sample of ISL images after preprocessing.

**Figure 4:** Architecture of proposed model.

**Figure 5:** Flow diagram of the proposed model.

**Figure 6:** Working of the proposed methodology.

**Figure 7:** (a): Scores of training dataset; (b) scores of testing dataset.

**Figure 8:** Comparison of the scores of the overall model.

**Figure 9:** Confusion matrix for 35 categories between actual and predicted values.

**Figure 10:** (a) Cross-entropy loss; (b) classification accuracy.

**Figure 11:** Working of WebRTC.

**Figure 12:** (a–c) The outcomes when person 1 contacts another person and the subtitles appear on the other person's calling screen.

**Table 1:** Results CNN and LSTM algorithms with proposed model.

Evaluation metric	CNN	LSTM
Accuracy	98.219	99.091
Precision	97.219	97.210
Recall	98.210	98.219
*F*1 score	92.323	92.347

## Data Availability

No data were used to support this study.
